The article "Genetic Multipartitions Based on D-Loop Sequences and Chromosomal Patterns in Brown Chromis, Chromis multilineata (Pomacentridae), in the Western Atlantic" was published in 2014. Journal: Biomed Res Int.

# Genetic Multipartitions Based on D-Loop Sequences and Chromosomal Patterns in Brown Chromis, *Chromis multilineata* (Pomacentridae), in the Western Atlantic

**DOI:** 10.1155/2014/254698

**Published:** 2014-10-19

**Authors:** Inailson Márcio Costa da Cunha, Allyson Santos de Souza, Eurico Azevedo Dias, Karlla Danielle Jorge Amorim, Rodrigo Xavier Soares, Gideão Wagner Werneck Félix da Costa, Erik García-Machado, Pedro Manoel Galetti, Wagner Franco Molina

**Affiliations:** ^1^Departamento de Biologia Celular e Genética, Centro de Biociências, Universidade Federal do Rio Grande do Norte, 59078-970 Natal, RN, Brazil; ^2^Centro de Investigaciones Marinas, Universidad de la Habana, Calle 16, No. 114, 11300 Habana, Cuba; ^3^Departamento de Genética e Evolução, Universidade Federal de São Carlos, Rodovia Washington Luís, Km 235, 13565-905 São Carlos, SP, Brazil

## Abstract

Connectivity levels among Brazilian reef fish fauna populations have attracted growing interest, mainly between mainland shores and oceanic islands. The Pomacentridae, whose phylogeographic patterns are largely unknown in the Atlantic, are a family of dominant fish in reef regions. We present data on the variability and population structure of damselfish *Chromis multilineata* in different areas along the northeast coast of Brazil and in the waters around the oceanic islands of Fernando de Noronha (FNA) and Saint Peter and Saint Paul Archipelago (SPSPA) through analysis of the HVR1 mtDNA sequence of the control region. The remote SPSPA exhibits the highest level of genetic divergence among populations. Conventional and molecular cytogenetic analysis showed similar karyotype patterns (2*n* = 48 acrocentrics) between these insular areas. Our estimates reveal three genetically different population groups of *C. multilineata* on the Brazilian coast. The level of genetic structure is higher than previous data suggested, indicating complex panel of interactions between the oceanic island and coastal populations of Brazil.

## 1. Introduction

Despite improvements in recent years, the aspects associated with dispersion, genetic variability, speciation, and evolution in fish populations distributed along the Brazilian coast and oceanic islands, for example, [1–6] continue to attract intense interest. This information is important to understanding the historical formation of current populations and their genetic divergence.

Among the typical species in sea reef environments are the Pomacentridae, one of the four most widely found families inhabiting tropical and subtropical reefs and one of the top 10 richest families in terms of diversity. It is the dominant group in number and diversity in most reef environments [7–9].

The article "Genetic Multipartitions Based on D-Loop Sequences and Chromosomal Patterns in Brown Chromis, Chromis multilineata (Pomacentridae), in the Western Atlantic" was published in 2014. Journal: Biomed Res Int.

On the Brazilian coast, the family Pomacentridae is represented by the genera* Abudefduf*,* Stegastes*,* Microspathodon*, and* Chromis* [7, 10]. The last genus contains about 75 species [7, 10–12], with* C. multilineata* dominant among pelagic holoplanktonic species [13–18]. The duration of the pelagic larval stage, an important biological characteristic involved in dispersion [19] and colonization, has been estimated to be between 24 and 33 days [18, 20, 21].

With amphi-Atlantic distribution, Brown chromis in the Western Atlantic extends from northern Florida to southern Brazil. It is one of the dominant species in insular regions, which show a sequential geographic position in relation to Brazil's Northeast coast, with different distances from the continent, such as the Rocas Atoll (267 km), Fernando de Noronha Archipelago (365 km), and the Saint Peter and Saint Paul Archipelago (1,100 km). More southward, it is found in the vicinity of Trindade Island and in the Meso-Atlantic region, in the waters around Ascension and Santa Helena islands [14–17].

Some reports involving fish populations of Fernando de Noronha Archipelago showed no evidence of genetic structuring in regard to the Northeastern coastal areas of Brazil [22]. In the Eastern Atlantic species of the genus* Chromis* with insular distribution have shown a pronounced divergence from a number of areas of the African coast. On the other hand, cytogenetic data of populations from Brazilian insular areas have largely improved [23, 24], showing homogeneity with coastal populations [25], and increased variation such as two* Caranx lugubris* karyomorphs in SPSPA [26] or conspicuous karyotype differences, revealing a new species of gobiid, in the FNA and Rocas Atoll [27].

The body of the species is greenish brown on the back and sides and white or silver on the abdomen, the edges of the dorsal and anal fins and the central part of the caudal fin tips are light yellow, while the edges of the dorsal fin are dark, often exhibiting a bright yellow spot immediately after the last ray of the dorsal fin [13]. However, semialbino individuals are described in the Saint Peter and Saint Paul Archipelago population [18]. This anomalous color pattern has been tentatively explained as a consequence of the isolation level of a small population of the species [21]. Previous analysis of mtDNA diversity in* C. multilineata* on a geographic macroscale (Greater Caribbean, Brazil, Meso-Atlantic region and Eastern Atlantic tropical coast) shows no genetic structuring between the Saint Peter and Saint Paul Archipelago and the Brazilian coast [28]. Although the cytogenetic patterns of this species have been previously reported for Brazilian coastal populations [29], the chromosomal aspects of insular populations remain unknown.

The article "Genetic Multipartitions Based on D-Loop Sequences and Chromosomal Patterns in Brown Chromis, Chromis multilineata (Pomacentridae), in the Western Atlantic" was published in 2014. Journal: Biomed Res Int.

Considering the evidence of gene flow restriction in marine organisms from oceanic islands in relation to the Brazilian coast [30–32], we show a more detailed analysis of the genetic connectivity level of Brown chromis populations between these regions, using HVR1 mtDNA. In addition, in order to identify cytotaxonomic markers for insular populations, classical cytogenetic techniques and double-FISH mapping of 18S and 5S ribosomal sequences were used. These data demonstrate a comprehensive panel of spatial genetic diversity distribution in* Chromis multilineata* and a variable relationship between insular and coastal populations.

## 2. Materials and Methods

### 2.1. Specimens, Collection Sites, and DNA Extraction

*Chromis multilineata* samples were collected by scuba diving in different Western Atlantic regions, encompassing coastal regions and oceanic islands in Brazil (Figure 1). A total of 14 individuals from Bahia: BA (12°55′S, 38°31′W); 25 from Rio Grande do Norte: RN (05°59′S, 34°59′W); 22 from Fernando de Noronha Archipelago: FNA (03°51′S, 32°26′W); and 14 from the Saint Peter and Saint Paul Archipelago: SPSPA (00°55′02′′N, 29°20′42′′W) were analyzed. Tissue samples (liver or pectoral fins) were preserved in 95% ethanol and stored at room temperature. Total DNA was isolated using phenol-chloroform extraction [33] and stored at 20°C. Some of the samples from insular regions were used to perform cytogenetic studies.

### 2.2. Amplification and Sequencing of HVR-1 mtDNA Sequences

The HVR-1 sequences of the D-loop region were amplified following the methodology proposed by Domingues et al. [35], using universal primers CR-A, 5′-TTCCACCTCTAACTCCCAAAGCTAG-3′ and CR-E, 5′-CCTGAAGTAGGAACCAGATG-3′ [36]. The polymerase chain reaction mix was composed of 10–50 ng of DNA mold; 1.5 mM MgCl_2_; 150 mM of dNTPs; 100 mM of buffer (Invitrogen, Tris-HCl and KCl, pH 7.8); 1.25 U of Taq polymerase (Gibco BRL); and 0.3 mM of each primer, with the addition of MilliQ water for a final volume of 25 *μ*L. The thermal cycling parameters were an initial denaturation step at 94°C for 2 min, followed by 35 cycles of 45 s and denaturation at 94°C, 45 s annealing at 52°C, and 1 min of extension at 72°C. Excess primers and dNTPs were removed with ExoSAP-IT (Amersham Pharmacia Biotech, Inc., UK). PCR products were sequenced on the Embrapa-Cenargen Sequencing Platform (Brasília/DF), with the BigDye Terminator v3.1 reaction kit, using the ABI 3130XL Genetic Analyzer (Applied Biosystems, Inc., Foster City, USA).

### 2.3. Nucleotide Sequence Analysis

The nucleotide sequences for the HVR1 region of mtDNA in* C. multilineata* were edited and checked through BioEdit 5.0.9 [37] and the automatic alignment of ClustalW was used, at a transversion/transition ratio of 0.2. Sequences of 312 pb were obtained and compared among individuals in different populations. Possible saturation between transitions and transversions was analyzed by Dambe [38]. Modeltest 3.7 [39] was applied to determine the most appropriate evolutionary model for nucleotide substitution found in the sequences. The neighbor-joining (NJ) tree for haplotype data was obtained through PAUP 4.0b10 [40]. Haplotype (h) and nucleotide (p) diversity were calculated in each site using Nei algorithms [41], while the fixation index (*F*_ST_) and molecular variance (AMOVA) were established using DnaSP 4b10.9 [42] and Arlequin 3.5 [43]. The Mantel test was performed to correlate genetic and geographic distances, in addition to determining the spatial pattern of genetic variation using Arlequin 3.5 [43].

The article "Genetic Multipartitions Based on D-Loop Sequences and Chromosomal Patterns in Brown Chromis, Chromis multilineata (Pomacentridae), in the Western Atlantic" was published in 2014. Journal: Biomed Res Int.

### 2.4. Specimens, Chromosomal Preparation, and Banding Procedures

Live individuals of* Chromis multilineata* from the Fernando de Noronha (*n* = 12) and Saint Peter and Saint Paul (*n* = 14) Archipelagos, including a semialbino specimen from the SPSPA, were used for cytogenetical characterization. All specimens were submitted to* in vivo* mitotic stimulation overnight by intramuscular inoculation with a complex of bacterial and fungal antigens [44]. Mitotic chromosomes were obtained via cell suspension from the anterior kidney [45]. Cell suspensions were dripped onto slides coated with a film of distilled water heated to 60°C. The diploid number was established by analyzing approximately 30 metaphases for each individual, after Giemsa staining. Given that the heterochromatin pattern of this species is known [29], specific heterochromatic regions were also analyzed using base-specific chromomycin A_3_ (CMA_3_) and 4′,6-diamidino-2-phenylindole (DAPI) fluorochromes [46], in superimposed sequential images of the same metaphase. The major ribosomal sites of the nucleolar organizer regions (NORs) and heterochromatin were identified in accordance with Howell and Black and Sumner [47, 48], respectively.

### 2.5. Probes for Chromosome Hybridization

The 5S and 18S rDNA probes, containing approximately 200 bp and 1400 bp, respectively, were obtained by PCR from the nuclear DNA of* Lutjanus analis* (Teleostei, Perciformes), using the primers A 5′-TAC GCC CGA TCT CGT CCG ATC-3′ and B 5′-CAG GCT GGT ATG GCC GTA AGC-3′ [49], NS1 5′-GTA GTC ATA TGC TTG TCT C-3′ and NS8 5′-TCC GCA GGT TCA CCT ACG GA-3′ [50], respectively. The former probe was labeled with biotin-14-dATP and the latter with DIG-11-dUTP, both by nick translation and in accordance with the manufacturer's specifications (Bionick Labelling System, Roche, Mannheim, Germany).

The article "Genetic Multipartitions Based on D-Loop Sequences and Chromosomal Patterns in Brown Chromis, Chromis multilineata (Pomacentridae), in the Western Atlantic" was published in 2014. Journal: Biomed Res Int.

### 2.6. Chromosome Hybridization

Fluorescence* in situ *hybridization (FISH) was performed on mitotic chromosome spreads [51] and dual-color FISH analysis was carried out using 5S rDNA and 18S rDNA probes. Briefly, the metaphase chromosome slides were incubated with RNAse (40 *µ*g/mL) for 1.5 h at 37°C. After denaturation of chromosomal DNA in 70% formamide (pH 7.0), the spreads were incubated in 2xSSC for 4 min at 70°C. Hybridization mixtures containing 100 ng of the denatured probe, 10 mg/mL dextran sulfate, 2xSSC, and 50% formamide (pH 7.0) in a final volume of 30 *µ*L were applied to the slides. Hybridization was conducted overnight at 37°C in a 2xSSC moist chamber. Posthybridization washes were carried out at 37°C in 2xSSC, 50% formamide (pH 7.0) for 15 min, followed by a second wash in 2xSSC for 15 min, and a final wash at room temperature in 4xSSC for 15 min. Signal detection was performed using avidin-FITC (Sigma, St. Louis, MO, USA) for the 5S rDNAprobe and anti-digoxigenin-rhodamine (Roche, Mannheim, Germany) for the 18S rDNA probe. Posthybridization washes were carried out in a shaker (150 rpm) and chromosomes were counterstained with DAPI (1.2 *µ*g/mL).

### 2.7. Image Processing

The slides were screened with an Olympus BX51 epifluorescence microscope and chromosomal plates were captured using a DP73 Olympus high resolution camera and CellSens© 1.9 Digital Imaging software. A total of 20–30 metaphases were analyzed for each specimen. Chromosome morphology was determined according to [52].

## 3. Results

### 3.1. Molecular Diversity

The sequencing of the amplified mtDNA HVR1 region of* C. multilineata* for each collection region produced partial sequences with 312 pb (GenBank accession numbers KM211594 and KM211689). Although the presence of tandem repetitions has been commonly described in a number of fish [53–56], they were not observed here. High haplotype and nucleotide diversity were observed in the samples (Table 1). A single haplotype (24), present in RN and SPSPA populations, was shared by all sampled regions. The composition of nucleotide bases showed A + T (65.85%) prevalence, in relation to C + G (34.15%).

### 3.2. Population Genetic Structure

The best evolutionary model determined for the sequences was TrN + I + G. The populations analyzed showed partially recognizable groups using the NJ method. Although tree topology has shown a number of branches with significant bootstrap values, most exhibit a mixture of individuals from different regions (Figure 2). Population structure matrices (A-F) analyzed by AMOVA (Table 2) indicate that most genetic variability is within populations. With a view to establishing the genetic divergence level of the SPSPA, its haplotypes were compared to different groups from other regions. In all cases, significant differences were identified (*P* < 0.05) in this insular region in relation to others (Table 3). *F*_ST_ values indicate structuring among the populations, especially in relation to the SPSPA (*F*_ST_ = 0.07–0.09), evidencing the presence of genetic structure. Coastal populations also showed structuring between each other. In fact, the RN population shows structuring in relation to BA (*F*_ST_ = 0.08, *P* < 0.05). The level of gene flow between sites, suggested by the number of migrants per generation (*N*_*m*_), showed *N*_*m*_ = 4.9 individuals between RN and SPSPA and unrestricted gene flow between RN and FNA (Table 3). The Mantel test showed no association between *F*_ST_ values and geographic distances (*P* > 0.05).

The article "Genetic Multipartitions Based on D-Loop Sequences and Chromosomal Patterns in Brown Chromis, Chromis multilineata (Pomacentridae), in the Western Atlantic" was published in 2014. Journal: Biomed Res Int.

### 3.3. Population Cytogenetic Traits

Samples of* C. multilineata *from the SPSPA and FNA had a karyotype with 48 acrocentric chromosomes (Figure 1). Ag-NORs were detected on the short arm of a medium-sized acrocentric chromosomal pair, previously defined by [29] as pair 8 (Figure 3(a), in the box). C-banding patterns were characterized by small centromeric blocks of heterochromatin on most chromosomes (Figure 3(b)). Fluorescent CMA_3_+/DAPI^−^ signals were identified exclusively on the nucleolar organizer regions (Figure 3(c), highlighted in the box). Mapping of 18S and 5S ribosomal sequences revealed a nonsyntenic location between these genes. The 18S rDNA sites were located on the short arms of pair 8, coincident with Ag-NORs regions, and 5S rDNA sites were located in an interstitial position on the short arm of pair 11 (Figure 3(d)). The semialbino individual from the SPSPA displayed similar chromosomal patterns to those of individuals from the FNA and SPSPA, including the position and frequency of 18S and 5S rDNA sites.

## 4. Discussion

The connectivity levels between populations of marine organisms are quite variable, and in some cases, evidence of pronounced genetic structure can be found [57], while in others, gene flow can be maintained even between long distances [58]. The geographic samples of* Chromis multilineata* show a high level of haplotypic diversity, with moderate genetic structure among the geographic regions analyzed. The broad haplotypic diversity is compatible with allopatric populations with a certain level of reproductive isolation in the recent past. Abrupt changes in ocean levels, caused by glaciation cycles during the Pleistocene, had a significant impact on coral reefs and the connectivity between their biotas [2, 59]. As a consequence of the alteration in habitat availability, these events caused demographic reductions and expansions, changing the level of contact and population distribution between geographic regions.

The article "Genetic Multipartitions Based on D-Loop Sequences and Chromosomal Patterns in Brown Chromis, Chromis multilineata (Pomacentridae), in the Western Atlantic" was published in 2014. Journal: Biomed Res Int.

In Atlantic species of* Chromis*, a number of genetic patterns indicate the influence of glacial events [35]. In* C. multilineata* this condition could have caused the diversity patterns observed, since it is distributed across a large number of geographic areas impacted by pleistocenic events [35, 60]. In different sampled regions, estimates obtained using Tajima's D [61] showed significant negative values (RN = −3.222; FNA = −3.147; BA = −3.256; SPSPA = −2.967; *P* < 0.0050), indicating an excess of low frequency polymorphisms, which, in historic demographic terms, suggests recent population expansions of the species. Geographic isolation cycles and secondary contacts are favorable for increased genetic diversity [62].

Previous population analysis in* C. multilineata* using mtDNA (cyt b) and involving geographic regions partially overlapping those covered by our study or in similar areas (SPSPA) showed an absence of population structure [28]. The more pronounced genetic structuring observed here, based on analysis of HVRI sequences, is possibly due to different molecular evolution rates between the mitochondrial sequences analyzed. In fact, the rapid evolution rate of HVRI sequences, roughly 25 times higher than that of cytochrome b [63], reveals more detailed information on long-dispersing species and that selective or demographic forces were recent events, as in* C. multilineata*.

The causes of genetic structure in reef environments may result from a historic interaction complex of different factors, such as physical connectivity between habitats, ocean currents, ecological patterns of species, larval behavior, and dispersal potential [59]. In general, the genetic differentiation between populations tends to increase with a decrease in the effective size of the population and with greater distance between samples [64]. Long geographic distances can increase genetic subdivision by restricting colonization events.

*Chromis multilineata* was genetically subdivided into three population groups in the sample areas of the Western Atlantic. The genetic profiles show one group composed of the SPSPA population, another formed by FNA and RN individuals, and a third by BA individuals (Figure 4). Population structure could be maintained by a combination of the geographic distances between regions and the action of Atlantic ocean currents, which act in a complex way due to variations in their force and direction throughout the year [34]. In this respect, the SPSPA, which is 1,100 km from the nearest point on the Brazilian coast and 1,824 km from the African coast, shows specific characteristics, contributing to its higher level of genetic divergence from other populations. In this oceanic region,* C. multilineata* exhibits significant genetic differentiation, both in relation to the most distant (*F*_ST_ = 0.092; *P* < 0.05) and nearest geographic locations (*F*_ST_ = 0.068; *P* < 0.05), such as the FNA (650 km). The genetic differences reported here indicate a genetic condition peculiar to this region, compared to Brazilian coastal areas.

The article "Genetic Multipartitions Based on D-Loop Sequences and Chromosomal Patterns in Brown Chromis, Chromis multilineata (Pomacentridae), in the Western Atlantic" was published in 2014. Journal: Biomed Res Int.

Haplotypic diversity and specific biological conditions classify the SPSPA as an evolutionarily independent geographic province. The exclusive genetic profile of the SPSPA population is reinforced by considerable biological evidence that highlights the effects of geographic isolation on connectivity. This includes the elevated level of endemism in many animal groups, such as mollusks, sponges (11.5%), and fish (8.3%) [30–32], which typifies a scenario of reduced gene flow with other oceanic regions. In addition, due to the high genetic variability present in this oceanic region, exclusive mutations and any selective role of this trait in local environmental pressures could explain adaptations in morphological characters and color variations [13, 33].

Interpopulation chromosomal analyses have been increasingly used in marine fish species with wide geographic distribution [23]. The data are used to identify population variations along the coast of Brazil [27, 65], between this region and the Caribbean [66], or to reaffirm differences between sister species [67]. In these cases, the changes observed involve primarily ribosomal subunits (Ag-NORs sites, 18S rDNA, and 5S rDNA sequences), which represent polymorphic chromosomal regions that reveal variations in their position and frequency.

In contrast to most Pomacentridae species, which show a numerically conserved karyotype of 48 chromosomes, with differences in the number of arms (NF = 48–90) [68, 69], Chrominae show a trend towards Robertsonian polymorphisms [29, 70]. Indeed, the reduction in chromosome number and presence of distinctive metacentric chromosomes in the Atlantic species* C. jubauna *and* C. flavicauda *result from centric fusions. Such specific polymorphisms are evidence of a transitory condition in Chrominae [57]. Robertsonian chromosomal rearrangements have been implicated in the origin of novel multiple sex chromosome systems in fish [71] and, in some cases, may contribute to the occurrence of genetically isolated populations.* Chromis multilineata*, on the other hand, shows a similar karyotype in all populations, on both the coast of Bahia [29] and the SPSPA and FNA.

The article "Genetic Multipartitions Based on D-Loop Sequences and Chromosomal Patterns in Brown Chromis, Chromis multilineata (Pomacentridae), in the Western Atlantic" was published in 2014. Journal: Biomed Res Int.

In the SPSPA, semialbinism has been observed in several* Chromis multilineata *individuals [16]. Albinism, semialbinism, and abnormal pigmentation in fish groups are rare genetic conditions in fishes [72–74]. Karyological data from specimens with abnormal coloration are scarce and limited to cultivated strains [75]. In marine fishes, cytogenetical analysis of* C. multilineata* from the SPSPA was the first survey performed in a natural population where semialbinism is recurrent. Although we performed classical cytogenetic procedures and the physical mapping of two ribosomal genes (18S and 5S rRNA), known polymorphic chromosome regions [76], the chromosomal patterns of the semialbino specimen showed no discernible chromosomal variation from the other individuals from insular populations.

Atypical body color variants may also be associated with extrinsic causes, such as pollution, dietary deficiency, and parasites [77–79]. However, the genetic differentiation of the SPSPA population does not rule out a genetic cause for the phenomenon. Exclusive occurrence of the* C. multilineata* semialbino phenotype in this area supports the occurrence of a larval autorecruitment process in this insular region.

Oceanographic conditions play an important role in the dispersion and colonization process in sea organisms, particularly in fish species that spend all their lives on reefs, where dispersion is restricted to the pelagic larval stage. Although the action of ocean currents is not the only factor that promotes dispersion of individuals in marine environments, their impact must always be considered. In the Tropical Atlantic the circulation of surface waters is complex and consists of an Equatorial gyre formed by North Equatorial Counter Currents (NECC), Guinea and three branches (north, central, and south) of the South Equatorial Current (SEC), which forms the North Brazil Current (NBC) and Brazil Current (BC) [34].

Even though the South Equatorial Current flows through the SPSPA towards the South American continent, a low gene flow from this region to other areas on the Brazilian coast was observed, especially to RN. In addition to distance, this finding could also be explained by the existence of larval retention around the islands. This hypothesis is plausible and in accordance with* C. multilineata* data.

Results of the numerical simulation of ocean circulation suggest an interaction between the Equatorial Current and the SPSPA [80]. This effect may decrease circulation velocity in areas adjacent to the SPSPA, in addition to generating a system of sublayer vortices which provide longer residence time in waters near the insular ecosystem. Thus, this condition expands the retention ability of organisms and nutrients, favoring recruitment mechanisms associated with the reproductive behavior of species that use the archipelago as a reproduction area. In fact, the occurrence of larval self-recruitment in the region has been suggested for many marine organisms that inhabit this insular region [81].

The article "Genetic Multipartitions Based on D-Loop Sequences and Chromosomal Patterns in Brown Chromis, Chromis multilineata (Pomacentridae), in the Western Atlantic" was published in 2014. Journal: Biomed Res Int.

Genetic patterns identified in* C. multilineata* are similar to those found in other Atlantic species of* Chromis*, analyzed by HVRI mtDNA sequences. In* C. limbata*, a drastic effect of Pleistocenic glaciation on genetic patterns was observed in the species [35]. This condition would have led to extinction or considerable population reduction in some regions, where surface water temperatures were critically low, and survival in less affected regions, which served as a refuge for the species [82]. Thus, the occurrence of recent population expansions in* C. multilineata* for all populations analyzed may be related to the same events.

Similarities in ichthyofauna allow dividing the Brazilian coast into two subgroups [83]. The first is formed by areas in the northern region and the Noronha Chain (a group of submerged mountains that are sequentially distributed toward the coast), whose emerged regions are formed by the Fernando de Noronha Archipelago and Rocas Atoll. The other subgroup has two branches, one formed by the northeast region, which includes RN, and the other by the Central region, which includes the Bahia coast, and the Southeast and Southern regions. In these areas a pattern of latitudinal genetic structure has been observed in a number of fish species.

The Brazilian continental shelf (2°S–8°S) is characterized by low temperature variation and high salinity variation, especially at the mouth of large rivers, such as the Amazon. Brazil's NE coast consists of a vast oligotrophic region, under the influence of Tropical Atlantic gyre circulation, including the north and south branches of the SEC, which flows westward to the Brazilian coast, where it bifurcates between 12° and 14°S (Bahia coast), forming the NCB to the north and CB to the south [34, 84]. Circulation patterns in the southern portion and the physical separation in the SEC, NCB, and CB could restrict wide gene flow between these regions [1]. Thus, biodiversity peculiarities in the northeast and central parts of the Brazilian coast suggest the simultaneous existence of patterns of adaptive divergence in RN populations (Northeast region) and BA (Central region), which may have contributed to the degree of genetic difference among populations of* C. multilineata* from these regions.

The article "Genetic Multipartitions Based on D-Loop Sequences and Chromosomal Patterns in Brown Chromis, Chromis multilineata (Pomacentridae), in the Western Atlantic" was published in 2014. Journal: Biomed Res Int.

## 5. Conclusion

*C. multilineata* shows a higher level of genetic structure than previous data suggested for this species along the Brazilian coast. Although all populations exhibit similar cytogenetical traits, unsuspected levels of genetic structure were identified among them. Indeed, some restrictions to gene flow are present between populations of the insular regions (FNA × SPSPA) and between coastal populations (RN × BA). The population of SPSPA exhibits a more conspicuous divergence from the others. These genetic variations suggest that they were established in recent times and indicate a complex scenario of interactions between populations of oceanic islands and those along the coast of Brazil.

## Figures and Tables

**Figure 1:** Collection sites of* C. multilineata*. Arrows indicate the main surface currents in the South Atlantic. BC: Brazil Current; sSEC: southern branch of the South Equatorial Current; cSEC: central branch of the South Equatorial Current; nSEC: northern branch of the South Equatorial Current; SSECC: South Equatorial Countercurrent; NBC: North Brazil Current, based on Lumpkin and Garzoli [34]. Highlighted in the box are* C. multilineata* individuals showing (a) normal color and (b) a semialbino pattern.

**Figure 2:** Neighbor-joining tree for D-loop sequences of* C. multilineata* individuals*. Lutjanus analis* was used as outgroup (^*^). Bootstrap values (>80%) are indicated on each node of the tree (1,000 pseudoreplicates). RN: Rio Grande do Norte; FNA: Fernando de Noronha Archipelago; BA: Bahia; SPSPA: Saint Peter and Saint Paul Archipelago.

**Figure 3:** Karyotypes of* C. multilineata* populations from Saint Peter and Saint Paul and Fernando de Noronha Archipelagos. Giemsa staining (a); C-banding (b); sequential CMA_3_/DAPI staining (c); and FISH-mapping (d) of 18S (red) and 5S (green) rDNA cistrons, respectively. The ribosomal sites corresponding to pairs 8 and 11 are highlighted in the boxes.

**Figure 4:** Spatial population genetic structure of* C. multilineata* based on partial sequences of HVR1 in the* D-loop* region. Population groups: I (I′, I′′), II, and III. BA: Bahia; RN: Rio Grande do Norte; FNA: Fernando de Noronha Archipelago; SPSPA: Saint Peter and Saint Paul Archipelago. The dotted lines delimit group I subpopulations; the solid line along the coast and islands indicates species distribution. The dotted lines represent moderate isolation between regions.

**Table 1:** Indexes of genetic diversity among sampled sites of *C. multilineata*.

Locality	*N*	Hn	Hd	*S*	ts	tv	*K*	П
RN	25	25	1.00	101	97	9	21.437	0.070
FNA	22	22	1.00	88	82	10	20.866	0.068
BA	14	14	1.00	81	73	13	22.714	0.073
SPSPA	14	14	1.00	74	66	18	24.011	0.078

Total	75	74	0.99	146	318	50	22.782	0.073

*N*: number of individuals, Hn: haplotype number, Hd: haplotype diversity, *S*: polymorphic sites, ts: transitions, tv: transversions, *K*: average of nucleotide differences, and *П*: nucleotide diversity.

The article "Genetic Multipartitions Based on D-Loop Sequences and Chromosomal Patterns in Brown Chromis, Chromis multilineata (Pomacentridae), in the Western Atlantic" was published in 2014. Journal: Biomed Res Int.

**Table 2:** Analysis of molecular variance (AMOVA) between *C. multilineata* collection sites with comparisons established between possible population groups ((A)–(F)).

Variation source	df	sd	% variation	*P*
(A) (RN + FN + BA) versus (SPSPA)				
Between populations	1	9.119	5.36	0.241
Between populations within groups	2	10.248	2.53	0.007∗
Within groups	71	235.523	92.10	0.000∗
Total	**74**	**254.891**		

(B) (RN + BA) versus (FNA + SPSPA)				
Between populations	1	17.966	−3.89	1.000
Between populations within groups	2	75.922	8.20	0.000∗
Within populations	71	1076.885	95.69	0.000∗
Total	**74**	**1170.773**		

(C) (RN + FNA) versus (BA) (SPSPA)				
Between populations	2	82.357	8.6	0.164
Between populations within groups	1	11.531	−0.95	0.635
Within populations	71	1076.885	92.35	0.000∗
Total	**74**	**1170.773**		

(D) (RN) versus (FNA)				
Between populations	1	11.531	−0.51	0.626
Within populations	45	589.171	100.51	
Total	**46**	**600.702**		

(E) (FNA) versus (SPSPA)				
Between populations	1	7.363	5.97	0.003∗
Within populations	34	120.026	94.03	
Total				

(F) (RN) versus (SPSPA)				
Between populations	1	42.869	9.22	0.000∗
Within populations	37	562.080	90.78	
Total				

(G) (BA) versus (SPSPA)				
Between populations	1	39.321	7.26	0.002∗
Within populations	26	487.714	92.74	
Total	**27**	**527.036**		

^*^Significant (*P* < 0.01).

**Table 3:** Fixation index *F*_ST_ (below diagonal) and migrant number (*N*_*m*_) in *C. multilineata* populations (above diagonal).

Population	RN	FNA	BA	SPSPA
RN		*∞*	5.093	4.925
FNA	−0.005		14.178	6.798
BA	0.089∗∗	0.034∗		6.385
SPSPA	0.072∗∗	0.068∗	0.092∗	

^*^ *P* < 0.05; ^**^ *P* < 0.001.
